# TACC3 as an independent prognostic marker for solid tumors: a systematic review and meta-analysis

**DOI:** 10.18632/oncotarget.20466

**Published:** 2017-08-24

**Authors:** June Wang, Shenlin Du, Wei Fan, Ping Wang, Weiqing Yang, Mingxia Yu

**Affiliations:** ^1^ Department of Clinical Laboratory & Center for Gene Diagnosis, Zhongnan Hospital of Wuhan University, Wuhan 430071, China; ^2^ Guangdong Provincial Key Laboratory of Medical Molecular Diagnostics, Guangdong Medical University, Dongguan 523808, China; ^3^ Department of Pathology, Zhongnan Hospital of Wuhan University, Wuhan 430071, China

**Keywords:** solid tumors, TACC3, survival, prognosis, meta-analysis

## Abstract

Recent studies have showed that the transforming acidic coiled coil 3 (TACC3), was aberrantly up-regulated in various solid tumors and was reported to be correlated with unfavorable prognosis in cancer patients. This study aimed to examine the relationship between TACC3 and relevant clinical outcomes. Pubmed, Web of Science, Embase and Cochrane Library were systematically searched to obtain all eligible articles. Pooled hazard ratios (HRs) and 95% confidence intervals (CIs) were calculated to evaluate the influence of TACC3 expression on overall survival (OS) and disease-free survival (DFS) in solid tumors patients. A total of 1943 patients from 11 articles were included. The result indicated that a significantly shorter OS was observed in patients with high expression level of TACC3 (HR=1.90, 95% CI=1.63–2.23). In the subgroup analysis, the association was also observed in patients with cancers of digestive system (HR=1.85, 95% CI=1.53–2.24). Statistical significance was also observed in subgroup meta-analysis stratified by the cancer type, analysis type and sample size. Furthermore, poorer DFS was observed in patients with high expression level of TACC3 (HR=2.67, 95% CI=2.10–3.40). Additionally, the pooled odds ratios (ORs) showed that increased TACC3 expression was also related to positive lymph node metastasis (OR=1.68, 95% CI=1.26–2.25), tumor differentiation (OR=1.90, 95% CI=1.25–2.88) and TNM stage (OR=1.66, 95% CI=1.25-2.20). In conclusion, the increased expression level of TACC3 was associated with unfavorable prognosis, suggesting that it was a valuable prognosis biomarker or a promising therapeutic target of solid tumors. Further studies should be conducted to confirm the clinical utility of TACC3 in human solid tumors.

## INTRODUCTION

Cancer is one of the major causes of death for its high morbidity and mortality, and it has become one of the major threats to global health [1]. WHO reports claimed that the number of new cancer cases in 2012 was 14.1 million, and in the same year, 8.2 million patients died of cancer and 32.6 million people living with cancers [2]. Although various therapeutic methods including surgery, chemotherapy as well as targeted therapy have made significant achievements, the 5-year-survival rate still remains unsatisfactory [3]. Thus, in order to help target care appropriately, it is vital to identify reliably prognostic biomarkers, guiding individualized treatment and improving unfavorable prognosis.

TACC3, derived from the transforming acidic coiled-coil proteins (TACCs) family contains a highly conserved C-terminal coiled-coil domain. It is encoded by the TACC3 gene which is located on 4p16.3, and is able to keep the centrosomal microtubules nucleation stable and regulate the integrity of centrosomes when mitosis occurs [4–6]. In addition to its role in mitosis, TACC3 has been proved to promote tumor growth. Knockdown of TACC3 inhibited the proliferation, invasion and tumorigenesis in renal cell carcinoma (RCC) cells [7]. Moreover, in several types of tumors, FGFR3–TACC3, a common TACC3 fusion gene, has been proved to promote the growth of cancer cells by promoting cell proliferation [8, 9].

Amounting researches have indicated that overexpression of TACC3 can be found in various solid tumors, such as lung cancer [10], ovarian cancer [11], glioblastoma [12], breast cancer [13], and hepatocellular carcinoma [14]. Further, a plenty of studies have showed that TACC3 overexpression was highly correlated with low survival rate in cancer patients [15–17]. However, single study may be not accurate and sufficient. Thus, it is necessary to gather relevant literatures and systematically analyze the clinical data for obtaining a better view of the potential clinical significance of TACC3 in solid tumor. In this study, we conducted this quantitative meta-analysis to clarify the relationship between overexpression of TACC3 and prognosis of solid tumors.

## RESULTS

### Study characteristics

The details of the literature retrieval process were presented in Figure 1. We searched 435 articles in the databases. After screening the titles and abstracts, 406 irrelevant or duplicate articles were excluded. Then because of no usable data, 18 papers were excluded. As a result, a total of 11 studies were enrolled for the final analysis [10, 14–23]. The main features of these eligible studies were displayed in Table 1. In total, the 11 studies provided a sample of 1,943 patients, with a minimum sample size of 79 and a maximum sample size of 237 patients. Because the cut-off definitions were various, the cut-off values were different in these studies. Among 11 studies, 9 were prospective cohort researches whereas 2 were retrospective. The major resources of literatures are from China (n=9), followed by South korea (n=1) and Korea (n=1). Moreover, there was one study in each of 7 types of cancer including breast cancer, colorectal cancer, gastric cancer, esophageal squamous cell carcinoma (ESCC), cholangiocarcinoma, prostate cancer, and glioma. And there were two studies in non-small cell lung cancer (NSCLC) and hepatocellular carcinoma (HCC). In all studies, there were 10 studies on OS, and 4 studies on DFS.

**Figure 1:** The flow diagram of the selection process in the meta-analysis

**Table 1:** Summary of all included eligible studies

First author	Year	Country	Number of patients	Tumor type	Stage	Method	Cut off	outcome	HR estimate	Nos
Song et al.	2015	China	203	Breast cancer	I-IV	ICH	IRS≥60%	OS	Reported	8
Zhou et al.	2015	China	237	Hepatocellular carcinoma	I-IV	ICH	≥0.04	OS DFS	Reported and Survival curve	8
Yun et al.	2015	China	186	Gastric cancer	I-III	ICH	IHC score≥50	OS DFS	Reported	7
Jiang et al.	2015	China	195	Non-small cell lung cancer	I-IV	ICH	score ≥6	OS	Reported	8
Nahm et al.	2015	South korea	188	Hepatocellular carcinoma	NM	ICH	-	OS	survival curve	8
Huang et al.	2014	China	209	Esophageal Squamous cell carcinoma	I-III	ICH	IRS≥60%	OS	Reported	7
Jung et al.	2005	Korea	163	Non-small cell lung cancer	I-III	ICH	-	OS	Reported	9
Du et al.	2015	China	161	Colorectal cancer	I-IV	ICH	IRS ≥ 5	OS DFS	Reported	8
He et al.	2016	China	79	Cholangiocarcinoma	I-IV	ICH	-	OS	Reported	7
Li et al.	2017	China	105	Prostate cancer	NM	ICH	SI≥6	DFS	Survival curve	9
Sun et al.	2017	China	217	Glioma	NM		-	OS	Reported	7

ICH: immunohistochemistry; IRS: immunoreactivity score; SI: staining index; NOS: Newcastle-Ottawa Scale; OS: overall survival; DFS: disease-free survival.

### Evidence synthesis

Ten studies reported the overall survival (OS) of eight types of cancer based on a total of 1838 patients’ different expression levels of ATCC3. The heterogeneity of these included studies was not significant (*I*^2^=0%, *P*=0.443). Therefore, the fixed-effects model was adopted to estimate the pooled hazard ratios (HRs) with corresponding 95% confidence interval (CI). As showen in Figure 2, the combined HR was 1.90(95% CI=1.63–2.23, *P*=0.000). Our analysis suggested TACC3 overexpression had a positive correlation with the worse overall survival in cancer patients.

**Figure 2:** Forest plot of HR for the correlation between TACC3 expression and overall survival (OS) in solid tumor

As shown in Table 3, further analyses of combined HR for OS were conducted. The pooled HRs of increased TACC3 expression on OS in patients with NSCLC, HCC and other cancers respectively were 2.02 (95% CI=1.37-2.96, *P*=0.000), 2.13 (95% CI=1.40-3.24, *P*=0.000) and 1.83 (95% CI=1.52-2.22, *P*=0.000). When we divided all cancer types into digestive system cancers and others, a similar result in digestive system cancers was found (HR=1.85, 95% CI=1.53-2.24, *P*=0.000).

**Table 3:** Subgroup meta-analysis of pooled HR for OS

Categories	No. of studies	No. of patients	Fixed-effects model		Heterogeneity	
			HR (95% CI) for OS	*P*-value	*I*^2^ (%)	*P*_*h*_
[1] OS	10	1838	1.90 (1.63-2.23)	0.000	0	0.443
[2] Cancer type						
1) Digestive system cancers	6	1061	1.85 (1.53-2.24)	0.000	37.7	0.155
Others	4	778	2.03 (1.53-2.68)	0.000	0	0.89
2) NSCLC	2	358	2.02 (1.37-2.96)	0.000	0	0.951
HCC	2	425	2.13 (1.40-3.24)	0.000	0	0.397
Others	6	1055	1.83 (1.52-2.22)	0.000	35.1	0.174
[3] Analysis type	8					
Survival curves	1	188	1.25 (0.34-4.63)	-	-	-
Multivariate	9	1650	1.92 (1.63-2.24)	0.000	6.2	0.383
[4] Sample size						
≥ 200	4	866	1.86 (1.48-2.34)	0.000	0	0.423
< 200	6	972	1.94 (1.56-2.41)	0.000	17.6	0.300

In addition, for OS, we stratified subgroup meta analysis in terms of analysis type and sample size, and demonstrated similar results in regard of the effects of upregulated TACC3 expression on OS.

### Increased TACC3 expression and DFS

There were just four studies which included 689 patients in total providing proper data for DFS analysis. Throughout these studies, we didn’t find serious statistical heterogeneity (*I*^2^=0%, *P*=0.625), meanwhile we analyze the pooled HRs with corresponding 95% CI by the fixed-effects model. The results indicated that TACC3 overexpression was positively associated the patients’ DFS in the enrolling studies (HR =2.67, 95% CI=2.10–3.40, *P*=0.000). Furthermore, the effects of TACC3 overexpression on DFS were consistent among different tumor types: hepatocellular carcinoma (HR=3.03, 95% CI=2.06-4.44), gastric cancer (HR=2.29, 95% CI=1.38-3.82), colorectal cancer (HR=2.05, 95% CI=1.13-3.72), and prostate cancer(HR=3.03, 95% CI=1.79-5.00) (Figure 3).

**Figure 3:** Forest plot of HR for the correlation between TACC3 expression and disease-free survival (DFS) in solid tumor

### TACC3 and clinical pathological factors

Another result was to explain the relationship between TACC3 expression and clinicopathological parameters (Figure 4). Five studies presented data about TACC3 expression was significantly associated with TNM stage (III-IV versus I-II OR=1.66, 95% CI=1.25-2.20, *P*=0.000, *I*^*2*^ =74.5%, *P*_*h*_ = 0.004), a pooled OR of 1.68 indicated a close relationship between increased TACC3 expression and lymph node metastases (N1/N2/N3 versus N0 OR =1.68, 95% CI=1.26–2.25, *P*=0.000, *I*^*2*^=55.5%, *P*_*h*_=0.061). No significant heterogeneity was observed, pooled estimates of 3 literatures showed that upregulated TACC3 expression was closely related to tumor differentiation (poorly versus well/moderately OR=1.90, 95% CI=1.25–2.88, *P*=0.003, *I*^2^= 0, *P*_*h*_=0.557).

**Figure 4:** Forest plots of odds ratios (OR) for the association between TACC3 overexpression and clinicopathological features in cancer patients **(A)** lymph node metastases; **(B)** TNM stage; **(C)** tumor differentiation.

### Sensitivity analysis

For testing the strength of our study, we performed a sensitivity analysis by alternately removing each study from the pooled analysis. The result were not obviously affected, indicating that our analyses should be reliable and stable (Figure 5).

**Figure 5:** Sensitivity analysis of the meta-analysis **(A)** Overall survival(OS). **(B)** Disease-free survival (DFS).

### Publication bias

The publication bias of included studies was estimated by Begg’s test. In the funnel plots, it showed there was no obvious asymmetry (Figure 6). And there was no evident publication bias for all the values of *P*>0.05.

**Figure 6:** Begg’s funnel plots for the studies involved in the meta-analysis of TACC3 expression and the prognosis of patients with solid tumors **(A)** Overall survival. **(B)** Disease-free survival. loghr, logarithm of hazard ratios; s.e., standard error.

## DISCUSSION

Though many studies have tried to explore how TACC3 plays a role in cancer progression, its potential molecular mechanisms of cancer progression remained unclear. In a study by Ma et al. [13], through elevating mRNA levels, TACC3 may promote invasive growth by elevated mRNA levels via the transition of breast cancer from ductal carcinoma *in situ* to invasive ductal carcinoma. Futhermore, EMT is a critical process in the early stage of the metastasis cascade and can be initiated by various signaling pathways. Recent researches have suggested that TACC3 is able to regulate epithelial-mesenchymal transition (EMT) of cervical tumor cells [24]. Besides, Hyoung et al. found that TACC3 utilize activating PI3K/AKT and extracellular regulated kinase (ERK) signaling pathways to help promote EMT process [25]. An important recent study demonstrated that TACC3 expression was downregulated by HDACIs and that targeted TACC3 knockdown suppresses CCA cell proliferation and colony formation [22]. TACC3 was also observed to contribute to the chemosensitivity in breast carcinoma cells [26–28] and NSCLC [10]. Knockdown of TACC3 can improve the sensitivity of tumor cells to chemotherapeutic drugs by effectively regulating premature senescence [27], and this suggests that TACC3 may be a potential biomarker for monitoring the efficacy of chemotherapy.

TACC3 has been identifed as a tumor-associated gene. Via changing key cell processes, initiating oncogenic signal transduction pathways and inducing genomic instability, the up- and downregulation of TACC3 may promote the development of cancers [29]. Most studies studies have demonstrated that TACC3 expression was upregulated in many cancers [30]. However, the downregulation of TACC3 expression was detected in ovarian and thyroid cancers [31, 32]. These differences in TACC3 expression between studies may be due to its different roles in various types of cancer. The high expression of TACC3 in cancers contributes to the proliferation, metastasis and invasion of tumors and may be a biomarker for cancer prognosis. In 2005, Jung *et al* revealed that a high expression of TACC3 could be considered as a negative prognostic factor for NSCLC patients and a prognostic indicator of poor survival rates [20]. Meantime, the increased expression of TACC3 was associated with extracapsular invasion in gastric cancer, which might be used as an independent predictor of shorter OS [18]. Therefore, we performed a meta-analysis to assess the association between high expression of TACC3 and prognosis of patients with solid tumors.

In our current meta-analysis, 11 studies consisting of 1943 patients was included. It was the first and most comprehensive meta-analysis systematically evaluating the prognostic value of TACC3 in patients with various tumors. Our studies reveals that there was a significant relationship between TACC3 overexpression and poor prognosis in cancer patients. Firstly, for OS, the pooled HRs results showed that increased expression level of TACC3 was associated with a shorter OS in solid tumor patients. Patients with high expression level of TACC3 have a short overall survival time than those with low TACC3 expression. It suggested that TACC3 could be an potential independent prognostic factor for predicting OS of cancer patients. In the stratified analysis for OS, patients with high levels of TACC3 may act as a reliable prognostic marker in digestive system cancers, which was concordant with our conclusion. Secondly, our data indicated that higher TACC3 expression suffered from poorer DFS. Taken together, TACC3 could serve as a promising biomarker for monitoring the progression of malignancies and represent a new target for the treatment of cancers.

Thirdly, we explored the clinicopathological significance of the expression levels of increased TACC3. The pooled data showed that increased TACC3 expression was positively associated with advanced clinical stage, lymph node metastasis and tumor differentiation, which indicated that upregulated TACC3 might have a significant relationship with advanced features of cancer. However, the degree of statistical heterogeneity in TNM stage and lymph node metastasis analysis were large, which may be due to the different types of cancer and cut-off values of TACC3 in the included studies.

Admittedly, there are several limitations in this meta-analysis. Firstly, majority of cases included in the meta-analysis were from China. Secondly, we estimated the HR and 95% CIs from the Kaplan–Meier survival curves in two studies, it might be less accurate than the data acquired directly from published statistics. Thirdly, the total sample size of the study is insufficient and 11 cancers cannot represent all types of malignancies. Finally, many included studies reported positive results because negative results would have little chance to be published. Therefore, our conclusions should be interpreted with caution. Larger-size and better design studies are needed to be implemented to confirm our results.

In summary, the overexpression of TACC3 is significantly associated with poor survival in patients with various types of cancer. It may be useful to act as a potential predictive marker of tumor prognosis and a promising therapeutic target for various cancer. However, considering the limited objectives of this meta-analysis, more standardized studies are needed to assess the findings.

## MATERIALS AND METHODS

### Study strategy

A systematic review of primary analysis was conducted according to the Preferred Reporting Items for Systematic Reviews and Meta-Analysis guidelines [33]. Pubmed, Web of Science, Embase and Cochrane Library were searched to obtain all relevant articles. The following search terms and all of their possible combination were used: (“cancer” OR “tumor” OR “tumour” OR “neoplasm” OR “carcinoma” OR “adenocarcinoma”) AND (“transforming acidic coiled coil 3” OR “TACC3”) AND (“prognosis” OR “prognostic” OR “outcome”). The search was performed up to May 1, 2017. References in relevant articles were also reviewed manually in case of the omission of any potentially relevant literature.

### Inclusion and exclusion criteria

Eligible studies included in this meta-analysis had to meet all of the following criteria: (1) Evaluating the association between TACC3 expression and prognosis of patients with any type of cancer; (2) Studies reporting survival data; (3) If the articles only provided survival curves without offering hazard ratios (HRs) and 95% confidence intervals (CIs) directly, appropriate data were extracted from the survival curves using Engauge Digitizer 4.1 software. (4) Studies published in English. (5) If there were duplicated data, we chose the most complete data or the most recent one. Exclusion criteria were as follow: duplicated studies; non-English papers; reviews articles; case reports; lack of original data; and non-human researches.

### Data extraction and quality assessment

Two reviewers (JEW and SLD) independently extracted information of all identified records according to pre-specified inclusion and exclusion criteria. The following data were extracted for each study: The first author’s name, publication year, country, number of patients, types of cancer, disease stage, detection method, cut off, outcome, HR estimate, score for TACC3 assessment. Data for OS and DFS were extracted from tables or Kaplan–Meier curves with respect to TACC3 expression [34, 35]. Any potential disagreements between the authors were resolved by discussions with a third reviewer(MXY). The Newcastle-Ottawa Scale (NOS) was applied to assess the methodological quality of all included studies [36]. According to the NOS criteria, all of the included studies got 7 scores or more are considered high quality articles (Table 2).

**Table 2:** Newcastle-Ottawa quality for included studies in this meta-analysis

Study	Selection			Comparability			Outcome			
	Representativeness of exposed	Selection of nonexposed	Ascertain-ment of exposure	No interest of study	Study design (cohort study)	Control for other confounding factors	Assessment of outcome	Follow-up time long enough (>5 years)	Adequacy number of follow-ups (>80%)	Total score
Song et al	1	1	1	0	1	1	1	1	1	8
Zhou et al.	1	1	1	0	1	1	1	1	1	8
Yun et al.	1	1	1	0	1	0	1	1	1	7
Jiang et al.	1	1	1	0	1	1	1	1	1	8
Nahm et al.	1	1	1	0	1	1	1	1	1	8
Huang et al.	1	1	1	0	1	0	1	1	1	7
Jung et al.	1	1	1	1	1	1	1	1	1	9
Du et al.	1	1	1	0	1	1	1	1	1	8
He et al.	1	1	1	0	1	1	1	0	1	7
Li et al	1	1	1	1	1	1	1	1	1	9
Sun et al	1	1	1	0	1	1	1	0	1	7

### Statistical analysis

Using the data collected from each eligible study, we performed the meta-analysis to evaluate the relationship between solid tumor’s TACC3 expression and patients’ prognosis. Pooled HRs and 95% CIs for two outcome endpoints (OS, DFS) were calculated via a fixed effects model or random effects model. The heterogeneity between studies was assessed with the Chisquare-based Q test and *I*^2^ statistics, and the *I*^2^ value indicated the degree of heterogeneity. A *P*-value ≤0.1 or *I*^2^≥50% indicated significant heterogeneity, in which case a random-effects model was used; if not, a fixed-effects model was used. Publication bias was estimated by Begg’s test, *P*<0.05 was considered statistically significant. We performed sensitivity analysis by omitting each study or specific studies to access the stability of the meta analysis results. Statistical analyses were conducted using Stata12.0 (Stata Corporation, College Station, TX, USA). All the *P*-values were determined by two-sided tests.
